The article "Analysis of Infertility Factors Caused by Gynecological Chronic Pelvic Inflammation Disease Based on Multivariate Regression Analysis of Logistic" was retracted in 2023. Reasons: unreliable results or conclusions; lack of ethics approval or compliance; concerns about the data; concerns about the peer review.

# Analysis of Infertility Factors Caused by Gynecological Chronic Pelvic Inflammation Disease Based on Multivariate Regression Analysis of Logistic

**DOI:** 10.1155/2022/7531190

**Published:** 2022-06-16

**Authors:** Linmei Liu, Gang Yang, Jigang Ren, Limei Zhang, Ting Wu, Qiao Zheng

**Affiliations:** ^1^Department of Traditional Chinese Medicine, Affiliated Hospital of North Sichuan Medical College, Nanchong, Jiangxi 637000, China; ^2^Department of Hepatobiliary Surgery, Affiliated Hospital of North Sichuan Medical College, Nanchong, Jiangxi 637000, China

## Abstract

In order to solve the complex and recurrent problem of chronic pelvic inflammation disease (CPID) in the process of the clinical treatment, a method of understanding the influencing factors of CPID by investigating the actual situation of clinical cases and using logistics regression analysis was proposed in this study. A total of 204 outpatients were selected from a certain hospital. The ratio of the cases in the experimental group to those in the control group stands at 1 : 1. The results were obtained as follows. According to the data of CPID patients collected in the paper, the majority of patients had a high school education background or below technical secondary school education background, accounting for 66.7%. And the majority of patients were manual workers, accounting for 69.1%. All the exp (*B*) values of the frequency of sex life per month ≥ 9 times, frequent sex life during menstruation, IUD contraception, no contraception, abortion ≥ 3 times, vaginal irrigation per week ≥ 1 time, and intrauterine surgery ≥ 3 times were more than 1. These seven factors were the risk factors for chronic pelvic inflammation. Oral contraceptives were a weak protective factor of chronic pelvic inflammation. These factors including early drug withdrawal (53.1%), without understanding the condition of the disease (35.7%), no time to review the disease (24.5%), and irregular medication (21.4%) accounted for a large proportion. They were associated with the recurrence of CPID. This method is aimed at providing some foundations for establishing effective prevention and control measures for chronic pelvic inflammation and providing a recognized clinical diagnosis and efficacy evaluation criteria for the treatment of chronic pelvic inflammation.

## 1. Introduction

Pelvic inflammatory disease (PID) refers to the inflammation of the female upper genital tract and its surrounding tissues, mainly including endometritis, salpingitis, fallopian tube and ovarian abscess, and pelvic peritonitis. Inflammation can be limited to one site or involve several sites simultaneously. Pelvic inflammation is divided into two categories, namely, acute and chronic. The deterioration of acute pelvic inflammation can cause diffuse peritonitis, sepsis, and septic shock. And it is life-threatening for severe cases. If it is not completely cured in the acute phase, it will become chronic pelvic inflammatory disease (CPID), which often lasts for a long time and occurs repeatedly. It can cause the diseases including infertility, tubal pregnancy, and chronic pelvic pain, seriously affecting women's health and increasing the economic burden of the family and society, as shown in Figure 1. Pelvic inflammation is a common gynecological disease. The main pathogens are staphylococcal, streptococcus, Escherichia coli, anaerobic bacteria, and so on [1]. In recent years, due to the wide prevalence of sexually transmitted diseases, the pathogen type of pelvic inflammatory disease has changed. And because of the change of modern human life patterns, the pathogenic factors of pelvic inflammatory disease have also become more complicated. At present, the incidence of pelvic inflammation has an upward trend, which has become the focus of domestic and foreign researches and has attracted the attention of experts from different countries. Because of the long disease course of PID that lasts for several months or years, or even decades, which has a great impact on women's health and fertility, the disease can lead to chronic pelvic pain (CPP), infertility, tubal pregnancy, and so on, seriously affecting women's health and increasing the economic burden of the family and society. Chronic pelvic pain caused by the long-term inflammation can cause a negative influence on women's daily life, work, and sexual life. It is because some viruses can threaten mother and child simultaneously through vertical infection that the treatment of PID is getting more and more attention and has become a highly anticipated topic in the medical community [2]. Over the years, professional workers have explored the etiology, pathogenesis, and treatment of pelvic inflammation unremittingly. Many drugs and methods have been used in the treatment of pelvic inflammation, but its curative effect is not very satisfactory. In order to explore the related factors of chronic pelvic inflammation and provide a scientific basis for further preventing the disease, the investigation of chronic pelvic inflammation still needs to be studied. This paper is aimed at investigating the related factors and relapse factors affecting the incidence of chronic pelvic inflammatory disease and at providing a reference for the prevention and treatment of this disease. At the same time, through the diagnosis of chronic pelvic inflammation patients and the exploration of the syndrome characteristics, it is aimed at providing new ideas for chronic pelvic inflammation syndrome and at providing clinical basis for scientific treatment [3]. Based on the above, logistic multivariate regression analysis was used to analyze the effect of chronic pelvic inflammation on infertility in women.

## 2. Literature Review

Pelvic inflammatory disease (PID) refers to a group of infectious diseases in the female upper genital tract, mainly including endometritis, salpingitis, fallopian tube and ovarian abscess (cyst), and pelvic peritonitis. Liu et al. believed that inflammation could be limited to one site and could also involve several parts at the same time. It could spread to the whole pelvic organs and peritoneum. The most common were salpingitis and salpingoophoitis, and simple endometritis and ovaritis were less common [4]. Reyftmann et al. believed that these symptoms including lower abdominal pain and discomfort, lumbosacral pain, low heat fluctuations, fatigue-prone, menstruation disorder, increased menstrual volume, and infertility were common. Even neurasthenia symptoms appeared, such as depression, fatigue and weakness, body discomfort, and insomnia [5]. Balla et al. believed that PID was the name of western medicine, and the name of pelvic inflammation did not appear in the ancient books of traditional Chinese medicine. According to the symptoms, signs, and clinical manifestations, it could be attributed to “female abdominal pain,” “leukorrhea disease,” “heat into blood room,” and “dysmenorrhea” [6]. Dabis considered that PID was one of the most frequent and important inflammation in pregestational women. PID was characterized by stubborn and recurrent disease, which seriously affects women's physical and mental health [7]. Chen et al. believed that its incidence rate remained high in recent years, and it was prone to recurrence, which seriously affected women's health. About 1 million women in the United States each year developed PID from a variety of pathogenic bacteria. The infection rate was highest among teenagers. Every year, more than 100,000 women were infertile due to pelvic inflammatory disease, and about 70,000 women have tubal pregnancy caused by PID [8]. According to Kaplan and Kirici, a woman spent 1060-3180 to treat PID in her lifetime on average. If the diagnosis and treatment were not timely, there would be a variety of sequelae, such as ectopic pregnancy, tubal ovarian abscess, infertility, dyspareunia, and chronic pelvic pain [9]. Siegenthaler et al. noted that chlamydial pelvic inflammatory disease had been reported as a risk factor for ovarian cancer. About 33.74% of PID patients were infected with HPV virus, so they were more prone to cervical cancer than the general population [10]. Yang et al. believed that the transmission route of pelvic inflammation usually included the following four forms: lymphatic system, blood circulation, spread along the genital mucosa, and direct spread. At present, it was believed that PID episodes were mostly related to the following factors: infection after intrauterine operation, sexual activity and age, lower reproductive tract infection, poor sexual hygiene, and inflammation of adjacent organs [11]. Lemly and Gupta summarized the following 10 inducing factors of PID: female genital anatomy characteristics, female genital natural defense function vulnerable, female life period of physiological characteristics, sexual activity, sexually transmitted diseases, contraception, abortion or vaginitis, vaginal flushing, iatrogenic infection, and other diseases such as tuberculosis and appendicitis [12]. Perhar et al. believed that the pathogens causing pelvic inflammatory disease had two sources, including aerobic and anaerobic pathogens from the original living in the vagina and pathogens from the outside, such as Neisseria gonorrhoeae, Chlamydia trachomatis, Mycobacterium tuberculosis, and Pseudomonas aeruginosa. The main pathogen was pyogenic bacteria, such as pathogens of streptococcus PID can be simple aerobe, simple anaerobic bacteria, or aerobic bacteria and anaerobic bacteria mixed infection, which may or may not be associated with sexually transmitted diseases. In order to prevent PID from attacking recurrently, in addition to the comprehensive treatment, attention must be paid to its nursing, so as to obtain better treatment effect and prevent its recurrence [13].

## 3. Research Methods

### 3.1. Diagnostic Criteria

Diagnostic criteria are formulated with reference to the relevant contents of the Guiding Principles for Clinical Research of New Chinese Medicine issued by the Ministry of Health.

(1) Medical history: having a history of acute pelvic inflammation
(2) Symptoms
  - Low fever and fatigue: systemic symptoms are not obvious. Sometimes the patients are prone to fatigue, with only low fever. Neurasthenia symptoms can appear for some patients with a long disease course, such as depression, physical discomfort, insomnia, and other diseases
  - Lower abdominal swelling pain or low lumbar swelling pain: this is the main clinical symptom. The pain is caused by the chronic inflammation of the uterus, tubal adhesion, or pelvic blood stasis. The pain may aggravate before and after fatigue, sexual intercourse, and menstruation [14]
  - Increased leucorrhea: leucorrhea is star-yellow or light yellow in form of water, or yellow green, sometimes with a bad smell
  - Menstrual imbalance: the symptom is with more menstruation volume or prolonged menstruation, due to pelvic blood stasis caused by chronic inflammation or affecting ovarian function
  - Infertility: the symptom appears due to tubal adhesion obstruction caused by chronic inflammation
(3) Signs: the uterus is often in a backward flexion position, with limited activity or fixed adhesion. When it is uterine myositis, the uterus can have tenderness. If it is salpingitis, the cord to phase the fallopian tube on one side or both sides of the uterus will be touched, with tenderness. If it is the fallopian tube water or fallopian tube ovarian cyst, cystic mass on pelvic side or both sides can be touched, with limited activity and tenderness. If it is pelvic connective tissue inflammation, the plate thickening can be touched on one or both sides of the uterus with tenderness. Or low ligament in the uterus is thickening and hardening, with tenderness [15].

For the above signs, the following two items should appear at the same time at least. The one is uterine movement being limited or adhesion fixation with tenderness. The other is tenderness in attachment area (corticulate thickening or sheet thickening or packing).

(4) Auxiliary examination
  - Blood routine: the total number of leukocyte or neutrophils slightly increases
  - Blood sedimentation rate examination: if inflammatory mass forms, the blood sedimentation rate increases slightly faster
  - B ultrasound examination: thickening fallopian tube, effusion, or pelvic inflammatory mass can be explored
  - Vaginal or cervical canal discharge smear examination: it is abnormal or pathogens can be detected
  - C reaction protein determination: if there is an inflammatory mass formation, examine whether C reaction protein increases or not
  - Serum CA-125 measurement: if there is an inflammatory mass formation, examine whether serum CA-125 increases or not
  - Laparoscopy: the formation of uterine and tubal adhesion lesions or pelvic inflammatory mass can be seen. It can be diagnosed according to the above main symptoms and necessary signs, combined with the medical history and auxiliary examination [16]

### 3.2. Data of the Experiment Subjects

A total of 204 outpatients were selected from a certain hospital. The ratio of the cases in the experimental group to those in the control group stands at 1 : 1. The control group was mainly selected from family members, relatives, friends, colleagues, or classmates of the selected cases. And healthy people aged no more than 3 years compared with the selected cases were randomly selected, with a total of 204 cases [17] (note: all research subjects had a sexual history).

The average age of the experimental group was 29.16 ± 7.63 years old. The average age of the control group was 30.08 ± 7.54 years old. There was no statistical difference in age between the two groups. Age distribution is shown in Table 1.

## 4. Results Analysis

### 4.1. Clinical Data of the Experimental Group

The minimum age was 19 years old, and the maximum age was 46 years old in the experimental group. And the patients were graded at 5 years as an age group. The specific information is shown in Figure 2.

As shown in Figure 2, in the collected data of CPID patients, the high incidence age of chronic pelvic inflammation was 25-34 years old, and the number of cases in this age group accounted for 55.9% of the total number of cases in the experimental group.

In the collected data of CPID patients, education and occupation are distributed in Figure 3.

As shown in Figure 3, in the collected data of the CPID patients, the majority of patients had a high school education background or below technical secondary school education background, accounting for 66.7%. And the majority of patients were manual workers, accounting for 69.1%.

### 4.2. Analysis of the Factors Associated with CPID Pathogenesis

By using the logistic regression analysis, the dependent variable *Y* is whether to suffer from chronic pelvic inflammation (0 = not suffer from CPID, 1 = suffer from CPID). The factors with the significant differences between the experimental group and the control group were obtained, including education, occupation, frequency of sex, menstrual sex, contraception (no contraception, IUD contraception, oral contraceptives), number of abortions, vaginal irrigation, intrauterine surgical operation, degree of work fatigue, and life pressure, which were regarded as independent variables. By using the backward deletion method, the binary logistic regression model was adopted. Logistic regression analysis was performed [18]. Results are shown in Table 2.

According to Table 2, the Sig. values of the eight factors listed were all less than 0.05, which were statistically significant. All the exp (*B*) values of the frequency of sex life per month ≥ 9 times, frequent sex life during menstruation, IUD contraception, no contraception, abortion ≥ 3 times, vaginal irrigation per week ≥ 1 time, and intrauterine surgery ≥ 3 times were more than 1. These seven factors were the risk factors for chronic pelvic inflammation. Combined with the regression factor *B* (positive correlation), it could be known that those with the above 7 factors were prone to chronic pelvic inflammation [19]. The exp (*B*) value of oral contraceptives was less than 1. Combined with the regression coefficient *B* (negative correlation), it indicated that it was a protective factor of chronic pelvic inflammatory disease. But its exp (*B*) value was close to 1, indicating that it was a weak protective factor.

The logistic regression equation was obtained from Table 2, as shown as follows:

(1) $$\begin{array}{c} P=\frac{e^{-1.194+0.691A+0.754B+0.311C+0.415D-0.023E+1.564F+0.761G+2.045H}}{1+e^{-1.194+0.691A+0.754B+0.311C+0.415D-0.023E+1.564F+0.761G+2.045H}}, \end{array}$$

where *A* is the frequency of sex life per month ≥ 9 times, *B* is the frequent sex life during menstruation, *C* is the IUD contraception, *D* is the no contraception, *E* is the oral contraceptives, *P* is the abortion ≥ 3 times, *G* is the vaginal irrigation per week ≥ 1 time, and *H* is the intrauterine surgery ≥ 3 times.

The positive probability of CPID can be calculated in the regression equation.

### 4.3. Analysis of the Factors Associated with the Recurrence of CPID

Among the 204 CPID cases investigated, 98 were patients with CPID recurrence. The recurrence patients filled in the recurrence-related factor table and the recurrence-related factors were investigated [20]. The results are shown in Table 3.

As can be seen from Table 3, according to the collected data in this survey, these factors including early drug withdrawal (53.1%), without understanding the condition of the disease (35.7%), no time to review the disease (24.5%), and irregular medication (21.4%) accounted for a large proportion. They were associated with the recurrence of CPID.

As shown in Table 4, in the collected data in this paper, the factor stopping the medication after the symptoms decrease by yourself (55.1%) accounted for a large proportion.

As can be seen from Table 5 that in the collected data in this survey, patients have a good compliance with doctors' advice on paying attention to hygiene and forbidding sex life during menstrual period, but poor compliance with regular review [21].

### 4.4. Discussions

As for patient care, patients suffering from CPID should follow the following five pieces of advice. First, one should pay attention to rest, avoid sex life being too frequent, and arrange the work and rest time. Second, one should adjust the mood to have a happy and optimistic spirit. Third, one should protect the spleen and stomach, pay attention to the diet and nutrition, and avoid spicy and stimulating foods. Fourth, one should beware of the invasion of wind, cold, and humid heat. Fifth, one should do appropriate exercises and strengthen the resistance ability of the body. Logistic regression is a multivariate analysis method to study the relationship between dichotomous or multicategorical dependent variables and multiple influencing factors. Logistic regression belongs to probabilistic regression, which is applicable to data with categorical variables (including ordered classification and disordered classification) [22]. According to the study design, it can be divided into nonconditional logistic regression and conditional logistic regression. According to the type of dependent variable, it can be divided into binary logistic regression, multiclassified disordered logistic regression, and multiclassified ordered regression. In dichotomy logistic regression, if the effect of an event (such as disease or not)*Y*(dependent variable) is affected by a group of independent variables*X*_1_, *X*_2_, *X*_3_, ⋯, *X*_*m*_that is dichotomized, the value of*Y* = 1indicates an event (such as disease and positive reaction), and*Y* = 0means an event does not occur (such as disease does not occur and negative reaction). Logistic regression analysis is widely used in the epidemiological study of disease risk factors and can also be used to screen the meaningful symptoms of syndrome differentiation. The syndrome is composed of a group of symptoms of different influences on the syndrome, which should distinguish between the primary and secondary symptoms. A logistic regression model of the syndrome can be established if the symptoms of the syndrome are used as the dependent variable *Y* and the symptoms appear in the syndrome are used as the independent variable *X*. The different contribution rates of these independent variables (symptoms) to the dependent variables (syndrome) can be analyzed by logistic regression. And the independent variables with too small or more scattered contribution rates can be excluded.

## 5. Conclusion

Chronic pelvic inflammation disease (CPID) is a common disease clinically in gynecology, which frequently occurs. The treatment of chronic pelvic inflammation is a more complex process. In this study, CPID was investigated with the help of the case-by-case method, and the related factors and recurrence characteristics of CPID were preliminarily understood.

The results of this study are shown as follows.

1. By the means of *X* and *X*^2^ test, the correlation factors of the difference with statistical significance between the experiment group and the control group were found. By using logistic regression analysis, the high risk factors of chronic pelvic inflammation were obtained including the frequency of sex life per month ≥ 9 times, frequent sex life during menstruation, IUD contraception, no contraception, abortion ≥ 3 times, vaginal irrigation per week ≥ 1 time, and intrauterine surgery ≥ 3 times. And the weak protective factor was oral contraceptives
2. According to the collected data in this survey, these factors including early drug withdrawal (53.1%), without understanding the condition of the disease (35.7%), no time to review the disease (24.5%), and irregular medication (21.4%) accounted for a large proportion. They were associated with the recurrence of CPID

## Figures and Tables

**Figure 1:** Influencing factors of pelvic inflammation.

**Figure 2:** Age distribution of the CPID cases.

**Figure 3:** The distribution of education and occupation of the CPID cases.

**Table 1:** The distribution of CPID cases and age of the control group.

Age (years old)	Case load (case)	The control group (case)
Below 20 (not including 20)	3	2
20-24	32	35
25-29	62	61
30-34	52	55
35-39	39	36
Above 40 (including 40)	16	15
Total	204	204

Note: the age distribution of the two groups was tested by *X*^2^. *P* > 0.05. It is not significant.

**Table 2:** Results of the logistic regression analysis of the factors associated with CPID.

Correlative factors	*B*	S.E.	Wald	df	Sig.	Exp (*B*)	95.0% C.I. for exp (*B*)	
							Lower	Upper
The frequency of sex life per month ≥ 9 times	0.691	0.297	5.430	1	0.020	1.996	1.116	3.570
Frequent sex life during menstruation	0.754	0.259	8.510	1	0.004	2.126	1.281	3.528
IUD contraception	0.311	0.140	4.914	1	0.027	1.365	1.037	1.796
No contraception	0.415	0.146	8.061	1	0.005	1.514	1.137	2.016
Oral contraceptives	-0.023	0.006	13.027	1	0.000	0.977	0.965	0.989
Abortion ≥ 3 times	1.564	0.774	4.084	1	0.043	4.778	1.048	21.783
Vaginal irrigation per week ≥ 1 time	0.761	0.771	0.976	1	0.032	2.141	0.473	9.700
Intrauterine surgery ≥ 3 times	2.045	0. 807	6.421	1	0.011	7.732	1.589	37.675
Constant	-1.194	0.338	12.450	1	0.000	0.303		

**Table 3:** Table of correlative factors related with recurrence of CPID.

Correlative factors	Number	Percentage (%)
No time to review the disease	24	24.5
Underestimating the disease	12	12.2
Without understanding the condition of the disease	35	35.7
Irregular medication	21	21.4
Early drug withdrawal	52	53.1
Other	8	8.2

Note: patients should fill in two or more related factors at the same time when filling in the form.

**Table 4:** Reasons for drug withdrawal.

Reasons	Number	Percentage (%)
Forgetting to take medicine	8	8.2
Stopping the medication after the symptoms decrease by yourself	54	55.1
Poor effect	16	16.3
The side effect of drug	9	9.2
High prices	11	11.2

**Table 5:** Table of the doctor's advice.

	Regular medication	Paying attention to hygiene	Regular review	Forbidding sex life during menstrual period
Yes	61.2	66.3	80.6	51.2
No	38.8	33.7	19.4	48.8

## Data Availability

The data used to support the findings of this study are available from the corresponding author upon request.
